# Association between Polymorphism of the Interleukin-13 Gene and Susceptibility to Hepatocellular Carcinoma in the Chinese Population

This article has been retracted.

**DOI:** 10.1371/journal.pone.0116682

**Published:** 2015-02-06

**Authors:** Yan Deng, Ming Xie, Li Xie, Jian Wang, Taijie Li, Yu He, Ruolin Li, Shan Li, Xue Qin

**Affiliations:** 1 Department of Clinical Laboratory, First Affiliated Hospital of Guangxi Medical University, Nanning, Guangxi, China; 2 Department of Medicine Research, First Affiliated Hospital of Guangxi Medical University, Nanning, Guangxi, China; University of North Carolina School of Medicine, UNITED STATES

## Abstract

**Objective:**

Interleukin-13 (IL-13) is a potent pleiotropic cytokine that is produced by activated CD4 T cells. This study was undertaken to determine the relationship between two IL-13 gene single nucleotide polymorphisms (SNP rs1800925 and SNP rs20541) and the incidence of hepatitis B virus-related (HBV) hepatocellular carcinoma (HCC).

**Method:**

Three hundred and ninety-eight HBV-positive individuals (192 HCC and 206 patients with chronic hepatitis) and one hundred and ninety-two healthy participants from the First Affiliated Hospital of Guangxi Medical University were enrolled in this study.

**Results:**

The results showed no significant differences between the genotype and allele frequencies of the IL-13 gene rs1800925 and rs20541 polymorphisms and chronic hepatitis B risk after adjusting for age, sex, tobacco use, and alcohol intake using binary logistic regression analyses. Regarding the rs20541 SNP, the GA genotype was significantly related to a decreased risk of HCC after adjusting for age, sex, tobacco use, and alcohol intake using binary logistic regression analyses (The odds ratio (OR) = 0.54, 95% confidence intervals (CI) 0.34–0.87). The adjusted OR for the GA and AA genotypes combined was 0.68 (95% CI 0.39–0.90).

**Conclusion:**

This study indicates that the functional IL-13 rs20541 polymorphism may contribute to the risk of HCC and that the rs20541 polymorphism is a protective factor for HCC.

## Introduction

Hepatocellular carcinoma (HCC) is one of the most common malignancies in humans. Epidemiologic evidence indicates that the main risk factor for HCC is hepatitis B virus (HBV). More than 80% of HCC cases are HBV-related [1]; however, the incidence of HCC in high-risk patients who were chronic HBV infected is only about 20% [2]. Other strong risk factors that contribute to the development of HCC have been well-documented and include exposure to aflatoxins, alcohol and tobacco abuse, and decreased intake of some antioxidant micronutrients [3,4]. Recently, several reports have shown that the occurrence and development of tumors such as HCC [5], breast cancer [6], gastric cancer [7], and pancreatic cancer [8] are associated with cytokine genes.

Interleukin-13 (IL-13) is a potent pleiotropic cytokine that is produced by activated CD4 T cells [9]. The beneficial effects of IL-13 include switching B cells to produce immune globulin E (IgE) and promoting the secretion of major histocompatibility complex (MHC) class II molecules. In addition, IL-13 can inhibit the production of inflammatory cytokines such as IL-1α, IL-4R, IL-8, and tumor necrosis factor (TNF)-α [10]. The human IL-13 is encoded by a gene located on chromosome 5q31 region and encompasses 2938 bps. Quiet a few single nucleotide polymorphisms (SNPs) have been identified for this gene. For example, IL-13 SNP rs20541 is a common coding SNP in exon 4, which is located at position 130 and resulted in a change from G to A. IL-13 SNP rs20541 has been reported to be associated with a decrease in the affinity of IL-13 for the IL-13 receptor and an increase in the expression of IL-13 in patients with asthma [11,12]. Rs1800925 is another common SNP of IL-13, located in the 5’ flanking region, which usually causes C to T substitution [13]. In addition, interindividual variation in the IL-13 polymorphism of rs1800925 may regulate the binding of STAT transcription factors，which have been reported to be related to alter the production of IL-13 in activated T cells [14].

Several genetic factors like IL-10, IL-18, and IL-12 have been confirmed to be involved in the development of antibodies to the HBV surface antigen in the case of hepatitis B vaccination or natural HBV transmission [15, 16]. It has been reported that through involvement in the T helper 1 / T helper 2 (Th1/Th2) system, the polymorphisms of IL-4R and IL-13 may consist as a common etiologic pathway in anti-HBs development [10]. The aim of this study was to uncover the relationship between the IL-13 gene SNP rs1800925 and SNP rs20541 polymorphisms and the incidence of HBV-related HCC.

## Materials and Methods

### Study population

398 HBV-positive individuals (192 HCC and 206 patients with chronic hepatitis) from the First Affiliated Hospital of Guangxi Medical University were enrolled in this study. The clinical criteria for HBV infection were confirmed by the criteria listed in our previous study [5]. The clinical criteria for chronic hepatitis B is defined by the elevation of alanine aminotransferase (ALT) (≥ 2 times the upper limit of normal reference) over a period of six months and HBV DNA level ≥ 1000 IU/mL. The diagnosis of HBV-related HCC was confirmed by computed tomography/ultrasound, magnetic resonance imaging (MRI), and laboratory tests. One hundred and ninety-two healthy participants were selected from the health center of the First Affiliated Hospital of Guangxi Medical University. The criteria for healthy participants was that they had no previous diagnosis of cancer or other serious illness and no family history of cancer or other serious illness. Written informed consent was obtained from all study participants. The study met the criteria of the Institutional Review Board of Human Research of the First Affiliated Hospital of Guangxi Medical University.

### DNA extraction and genotyping of the SNPs

Fresh blood samples were collected in EDTA-containing tubes. Genomic DNA was extracted using a QIAamp DNA blood mini kit (QIAGEN GmbH, Hilden, Germany) as instructed by the manufacturer. The analysis of IL-13 polymorphisms rs1800925 and rs20541 was performed by the classic polymerase chain reaction restriction fragment length polymorphism (PCR-RFLP) method. The accuracy of the genotyping results was assessed using the ABI PRISM 3730 to examine the representative PCR-amplified DNA samples (Figs. 1 and 2). The two SNP primer sequences and the necessary reaction condition are listed in Table 1.

**Fig 1:** rs1800925 genotyping by direct sequencing: (a) CC genotype; (b) CT genotype; (c) TT genotype.

**Fig 2:** rs20541 genotyping by direct sequencing: (a) GG genotype; (b) GA genotype; (c) AA genotype.

**Table 1:** Primer sequence and the reaction condition for genotyping IL-13 polymorphisms.

Polymorphism	Primer sequence	Annealing temperature (C°)	Restriction enzyme	Product size (bp)
rs1800925	F: 5′-GGTTTCTGGAGGACTTCTAGGTA-3′	66°	Hpy8I	CC: 98bp+43bp TT: 141bp
	R: 5′-GCAGAATGAGTGCTGTGGAG-3′			CT: 141bp+98bp+ 43bp
rs20541	F: 5′-TGCTTTCGAAGTTTCAGTGGA-3′	62°	NlaIV	GG: 105bp+41bp AA: 146bp
	R: 5′-CATGTCCGAGACACCAAAATC-3′			GA: 146bp+105bp+41bp

### Statistical methods

The analysis of variance (ANOVA) method was used to evaluate the differences in demographic and clinical data among the groups. To test for deviations from the Hardy—Weinberg equilibrium, a χ^2^ test was used to compare the true genotype frequencies in the study to the expected ones among the subjects. Binary logistic regression was used for calculating the relative risk of each SNP, controlling for age and gender as covariates. OR and their 95% CIs were obtained as measures of association and precision between polymorphism genotypes. Dominant models were adopted for calculating odds ratios to assess the effect of an SNP variant. All statistical analyses were performed using the SPSS software, version 13.0. All statistical tests were two-sided and the statistical significance was set at *p* < 0.05.

## Results

Detailed patient demographics for all groups including gender, age, tobacco use, education, and alcohol intake are listed in Table 2. The genotype frequencies of each of the IL-13 gene polymorphisms were categorized into groups, as shown in Table 3. The mean age of the control group patients was 44, the mean age of the chronic hepatitis B patients was 47, and the mean age of the HBV-related group patients was 47. The results showed no significant difference in age among the three groups. As for gender distribution, there was a significant difference among the three groups (p = 0.00). Education, tobacco use, and alcohol intake did not differ significantly among the control, chronic hepatitis B, and HBV-related groups (p = 0.25, p = 0.15, and p = 0.09, respectively). Furthermore, we tested the Hardy-Weinberg equilibrium (HWE) for the two selected SNPs. The distribution of the rs1800925 and rs20541 SNPs among the controls was consistent with the HWE test (p = 0.51 and p = 0.91, respectively).

**Table 2:** Characteristics of study subjects.

Groups	Healthy controls (n = 192)	Chronic hepatitis B patients (n = 206)	HBV-related HCC patients (n = 192)	P
Gender (M/F)	150/42	136/70	158/34	0.00
Age (yrs) (Mean±SD)	44.28±13.02	47.9±11.92	47.46±12.23	0.58
Education (yrs)	12.5 (±2.8)	12.3 (±2.0)	11.8 (±2.5)	0.25
Smoking status (%) (n)				0.15
Current	51.0 (98)	50.5（104)	56.3 (108)	
Past	23.4 (45)	30.1（62)	27.6 (53)	
Never	25.6(49)	19.4（40)	16.1 (31)	
Drinking (%) (n)				0.09
Current	46.8（90)	50.0（103)	53.1（102)	
Past	34.9（67)	29.5（61)	36.0（69)	
Never	18.3（35)	20.5（42)	10.9（21)	

**Table 3:** Genotype and allele frequencies of two SNPs in the IL-13 gene between HBV-related HCC patients and healthy controls.

Polymorphisms	Healthy controls	Chronic hepatitis B patients			HBV-related HCC patients		
	n = 192(%)	n = 206 (%)	*OR*(95%CI)*	*p* *	n = 192 (%)	*OR*(95%CI) *	*p* *
rs1800925							
Genotypes							
CC	128(66.6)	140(67.9)	1.00		122（63.5)	1.00	
CT	61 (31.8)	61(29.7)	0.87(0.46–2.32)	0.689	67 (34.9)	0.89（0.58–1.36)	0.586
TT	3 (1.6)	5(2.4)	0.81(0.39–2.01)	0.706	3 (1.6)	0.94（0.18–4.83)	0.945
C Allele	317(82.6)	341(82.8)	1.00		311(81)	1.00	
T Allele	67(17.4)	71(17.2)	0.92(0.56–1.37)	0.962	73(19)	0.91（0.63–1.32)	0.631
Dominant model							
CC	128(66.6)	140(67.9)	1.00		122(63.5)	1.00	
CT+TT	64(33.4)	66(32.1)	0.83(0.55–1.24)	0.355	70(36.5)	0.85(0.55–1.24)	0.752
rs20541							
Genotypes							
GG	68(35.4)	83(40.3)	1.00		46(24.0)	1.00	
GA	96(50.0)	85(41.2)	0.69(0.52–1.23)	0.408	117(60.9)	0.54（0.34–0.87)	0.015
AA	28(14.6)	38(18.5)	1.21(0.44–2.13)	0.512	29(15.1)	0.66（0.35–1.26)	0.211
G Allele	232(60.4)	251(60.9)	1.00		209(54.4)	1.00	
A Allele	152(39.6)	161(39.1)	0.95(0.65–1.32)	0.948	175(45.6)	0.78（0.59–1.05)	0.106
Dominant model							
GG	68(35.4)	83(40.3)	1.00		46(24.0)	1.00	
GA+AA	124(64.6)	123(59.7)	0.58(0.54–1.19)	0.319	146(76)	0.68(0.39–0.90)	0.023

*Adjusted for age, sex, smoking, and drinking when compared with the healthy controls

### Chronic hepatitis B patients versus healthy controls

The genotype and allele frequencies of IL-13 gene polymorphisms among the chronic hepatitis B patients and the healthy controls are shown in Table 3. In the chronic hepatitis B patients, the frequencies of the CC, CT, and TT genotypes of rs1800925 were 67.9%, 29.7%, and 2.4%, respectively, and in the healthy controls, they were 66.6%, 31.8%, and 1.6%, respectively. In the chronic hepatitis B patients, the frequencies of the GG, GA, and AA genotypes of rs20541 were 40.3%, 41.2%, and 18.5%, respectively, and in the healthy controls, they were 35.4%, 50.0%, and 14.6%, respectively. No significant effects were observed between the genotype and allele frequencies of the IL-13 gene rs1800925 and rs20541 polymorphisms and chronic hepatitis B risk after adjusting for sex, age, tobacco use, and alcohol intake using binary logistic regression analyses.

### HBV-related HCC patients versus healthy controls

The genotype and allele frequencies of the IL-13 gene polymorphisms among the HBV-related HCC patients and healthy controls are shown in Table 3. Using subjects with the CC genotype as a reference group, the results showed that there were no significant differences between the genotype and allele frequencies of the IL-13 gene rs1800925 polymorphisms and HCC risk after adjusting for sex, age, tobacco use, and alcohol intake using binary logistic regression analyses. Regarding the rs20541 SNP, we found a significant relationship between the rs20541 SNP and the risk of HCC (Table 3). Compared with the GG genotype, the GA genotype (but not the AA genotype) was significantly related to a decreased risk of HCC after adjusting for age, sex, tobacco use, and alcohol intake using binary logistic regression analyses (OR = 0.54, 95% CI 0.34–0.87). Adjusted OR for the GA and AA genotypes combined was 0.68 (95% CI 0.39–0.90).

### Stratified analysis

We next investigated whether the differences of genotype and allele frequencies were related to gender. Significant differences in the distributions of the IL-13 gene polymorphisms between HBV-related HCC patients and control groups were observed (Table 4). Men who carried the IL-13 (rs20541) GA genotype were associated with a decreased risk of HCC compared with patients carrying the GG genotype (OR = 0.53; 95% CI 0.32–0.90).

**Table 4:** Stratification analysis of IL-13 polymorphisms in healthy controls and HBV-related HCC patients.

	Male				Female			
Polymorphisms	Healthy controls	HBV-related HCC patients			Healthy controls	HBV-related HCC patients		
	n = 150(%)	n = 158(%)	*OR*(95%CI)*	*p* *	n = 42 (%)	n = 34 (%)	*OR*(95%CI)*	*p* *
rs1800925								
Genotypes								
CC	104(69.3)	100(63.3)	1.00		24(57.1)	22(64.7)	1.00	
CT	45(30.0)	56(35.4)	0.81(0.50–1.31)	0.392	16(38.1)	11(32.4)	1.33(0.51–3.49)	0.561
TT	1(0.7)	2(1.3)	0.50(0.05–6.09)	0.606	2(4.8)	1(2.9)	1.80(0.15–21.3)	0.643
C Allele	253(84.3)	256(81.0)	1.00		64(76.2)	55(80.9)	1.00	
T Allele	47(15.7)	60(19.0)	0.83(0.54–1.26)	0.372	20(23.8)	13(19.1)	1.32(0.60–2.93)	0.494
rs20541								
Genotypes								
GG	54(36.0)	37(23.4)	1.00		14(33.3)	9(26.5)	1.00	
GA	76(50.7)	95(60.1)	0.53(0.32–0.90)	0.025	20(47.6)	22(64.7)	0.79(0.28–2.24)	0.665
AA	20(13.3)	26(16.5)	0.55(0.44–1.13)	0.101	8(19.1)	3(8.8)	1.78(0.36–8.94)	0.481
G Allele	184(61.3)	169(53.5)	1.00		48(57.1)	40(58.8)	1.00	
A Allele	116(38.7)	147(46.5)	0.73(0.53–1.01)	0.065	36(42.9)	28(41.2)	1.08(0.57–2.07)	0.816

*Adjusted for age, smoking, and drinking when compared with the healthy controls

The frequencies of genotype and allele of these two SNPs in our control group were compared with those from the Haplotype Map (HapMap) Project (http://www.ncbi.nlm.nih.gov/snp/). Table 5 shows the differences between polymorphisms in healthy controls in the present study and other ethnicities’ healthy controls included in the HapMap project. For rs1800925 and rs20541 polymorphisms, the frequencies of allele in YRI (Yoruba in Ibadan) are significantly different from those in the present study. In the rs20541 site, there is a significantly lower detection rate of the CC allele (35.4%) in our data comparison with JPT (Japanese in Tokyo) and CEU (Utah residents with northern and western European ancestry) (51.2% and 60.2%, respectively). However, there were no significant differences in the two SNPs between the present study and CHB (Chinese Han in Beijing), with the exception of the G and A alleles of rs20541.

**Table 5:** Comparison of genotype and allele frequencies in the healthy control subjects of the present study with examples from the HapMap project.

Polymorphisms	Samples, N	Genotype frequency, n (%)			P values	Alleles frequency, n (%)		P values
rs1800925		CC	CT	TT		C	T	
Prensent Study	192	128(66.6)	61(31.8)	3(1.6)		317(82.6)	67(17.4)	
CHB	90	64(71.1)	24(26.7)	2(2.2)	0.65	152(84.4)	28(15.6)	0.58
JPT	72	54(75.0)	16(22.2)	2(2.8)	0.58	124(86.1)	20(13.9)	0.33
CEU	120	80(66.7)	34(28.3)	6 (5.0)	0.19	194(80.8)	46(19.2)	0.59
YRI	120	30(25.0)	64(53.3)	26(21.7)	0.00	124(51.7)	116(48.3)	0.00
rs20541		GG	GA	AA		G	A	
Prensent Study	192	68(35.4)	96(50.0)	28(14.6)		232(60.4)	152(39.6)	
CHB	86	42(48.8)	36(41.9)	8(9.3)	0.09	120(69.8)	52(30.2)	0.03
JPT	172	88(51.2)	66(38.4)	18(10.5)	0.01	242(70.3)	102(29.7)	0.01
CEU	226	136(60.2)	82(36.3)	8(3.5)	0.00	354(78.3)	98(21.7)	0.00
YRI	226	158(69.9)	56(24.8)	12(5.3)	0.00	372(82.3)	80(17.7)	0.00

HapMap, Haplotype Map; CHB, Chinese Han in Beijing, China; JPT, Japanese in Tokyo, Japan; CEU, Utah residents with northern and western European ancestry; and YRI, Yoruba in Ibadan, Nigeria

### Haplotype analysis

Table 6 shows the haplotype distribution in HCC patients and healthy controls. The haplotype comprised of the C allele of rs1800925 and the A allele of rs20541 was significantly associated with an increased risk of HCC (OR = 1.612, 95% CI 1.047–2.481). In contrast, the haplotype comprised of the rs1800925 T allele and the rs20541 G allele was associated with a significantly decreased risk of HCC (OR = 0.472, 95% CI 0.243–0.915). The remaining haplotypes were not associated with HCC.

**Table 6:** Haplotype distribution in patients with HCC and healthy controls.

Haplotype	HCC(%)	Healthy controls(%)	OR	P
CA	0.301	0.294	1.035	0.827
CG	0.509	0.532	0.913	0.526
TA	0.154	0.102	1.612	0.029
TG	0.036	0.073	0.472	0.023

## Discussion

In this study, we performed a large case-control study that determined the association between SNPs in the IL-13 gene and the presence of chronic hepatitis B and HBV-related HCC. The rs1800925 CT and TT genotypes were not associated with risk in either the chronic hepatitis B patients or the HBV-related HCC patients. Although the IL-13 rs20541 SNP does not appear to have a significant association with the risk of chronic hepatitis B, we found a significant relationship between the rs20541 SNP and the risk of HCC. The GA genotype of the rs20541 SNP, with a 50% frequency among controls, was significantly related to a decreased risk of HCC. Men who carried the IL-13 (rs20541) GA genotype were associated with a decreased risk of HCC compared with patients carrying the GG genotype. It is universally acknowledged that the IL-13 genetic background may be different from other individuals, we compared the genotype and allele frequencies of the two SNPs in our control group with those in different ethnicities from the HapMap. The results showed that the distribution of the two SNPs in the present study was similar to that in the CHB controls. However, when compared with YRI or European populations, it was significantly different, thus suggesting that the distribution of IL-13 gene frequencies might vary among different ethnic groups. Haplotype analyses showed a protective association between the haplotype tagged by the ‘no-risk’ alleles of the rs1800925 and rs20541 SNPs (TG haplotype). Meanwhile, the same ‘no-risk’ alleles of the rs1800925 and rs20541 SNPs (CA haplotype) were significantly associated with increased risk of HCC.

IL-13 is well known as a Th2 anti-inflammatory cytokine that is involved in mediating B cell and mast cell proliferation and correlates with IgE synthesis, which is a major regulator in Th2-mediated disease [17]. Based on the key roles of IL-13 in the IgE pathway, a large number of genetic studies have focused on the contribution of IL-13 polymorphisms to the risk of allergic rhinitis and asthma. Bottema et al. [18] investigated IL-13 polymorphisms in rhinitis and asthma populations; their results showed that IL-13 rs1800925 was significantly associated with rhinitis, while the polymorphisms of rs20541 and rs1295685 were consistently associated with asthma and serum IgE, which were consistent with the results of haplotypes. A meta-analysis down by Lin et al. [19] exerted a tremendous fascination on the association between the polymorphisms of rs20541 and rs1800925 in the IL-13 gene and asthma, and the results demonstrated that the two polymorphisms are associated with a significantly increased risk of asthma. Evidence indicating that the IL-13 rs20541 SNP is associated with an increased risk of allergic rhinitis was reported by Ying et al. [20], who performed a meta-analysis that included 2,153 cases and 3,931 controls. To date, many epidemiological studies have been carried out to evaluate whether polymorphisms in IL-13 contribute to an individual’s susceptibility to cancer. Sun et al. [21] observed that IL-13 rs20541 GA and AA variant genotypes were significantly associated with a reduced risk of glioma (OR = 0.85, 95% CI 0.75–0.970). The IL-13 rs1800925 polymorphism was significantly associated with decreased a risk of glioma (CT vs. TT: OR = 0.72, 95% CI 0.55–0.93; CT/TT vs.TT: OR = 0.76, 95% CI 0.62–0.89) [22]. Patients harboring the IL-13 rs20541 T allele had a reduced risk of colorectal cancer [23]. In contrast, Hall et al. [24] reported that tobacco smokers in the Chinese population who were carriers of the IL-13 rs1800925 CT variant genotype had a 2.57-fold increased risk of bladder cancer. To the best of our knowledge, this is the first study documenting the relationship between IL-13 genetic variants and HCC.

The body’s immune response to hepatitis B and C infections, viral clearance, and inflammation have been implicated in cancer diagnosis, prognosis, and therapy [25, 26]. IL-13 is a crucial anti-inflammatory and immunomodulatory factor that can trigger cancer-directed immunosurveillance [27]. IL-13 has been reported to be overexpressed in a majority of glioma cell lines and glioblastoma tumor tissues [28]. In addition, through the IL-4R signaling pathway, IL-13 plays a key role in downregulating tumor immunosurveillance, and in the process of cancer immunotherapy through inhibiting of IL-13 have been proven to be a benificial tool [29]. Terabe et al. [30] hold the view that a decrease in IL-13 production was associated with a lower recurrence of tumors. Furthermore, in human glioma cell lines, experiments by Liu’s group have recently shown that IL-13 could inhibit proliferation of low-grade glioma [31]. Skinnider et al. [32] found that IL-13 plays an important role in stimulating the growth of the Reed-Sternberg cell, which can inhibit tumor immunosurveillance through the signal transducer and activator of transcription (STAT) 6 in Hodgkin’s disease. Our study indicates that the IL-13 rs20541 SNP is a protective factor for HCC, although the functional relevance of the IL-13 rs20541 SNP is not completely understood.

In conclusion, our study provides evidence that the functional IL-13 rs20541 polymorphism may contribute to the risk of HCC. However, the results of this paper were obtained with a relatively limited sample size and single ethnic population. Therefore, larger studies of other ethnic populations, especially studies of the combined effects of the gene-gene and gene—environment are needed to confirm the current results.
